# Comparison of Bacterial and Fungal Community Structure and Potential Function Analysis of Yak Feces before and after Weaning

**DOI:** 10.1155/2022/6297231

**Published:** 2022-08-30

**Authors:** Yuanyuan Li, Xin Li, Yanfeng Liu, Cunxi Nie, Cheng Chen, Junli Niu, Wenju Zhang

**Affiliations:** ^1^College of Animal Science and Technology, Shihezi University, Shihezi, Xinjiang 832000, China; ^2^College of Life Sciences, Shihezi University, Shihezi, Xinjiang 832000, China; ^3^Feed Research Institute of Xinjiang Academy of Animal Sciences, Ürümqi, Xinjiang 830000, China

## Abstract

Weaning is one of the most stressful periods in yak growth. However, the impact of weaning on microbial diversity, structure, and potential function of yak feces is not clear. In this study, 12 Xinjiang yaks aged 3, 4, 5, and 6 months old were selected to collect fresh feces before and after weaning. Through 16S rRNA and ITS high-throughput sequencing, the dynamic distribution and potential function of yak fecal, bacterial, and fungal communities in each month were revealed. The study found that the richness of fungi had a significant impact on weaning. At the phylum level, *Firmicutes*, *Bacteroidetes*, *Ascomycota*, and *Basidiomycota*, and at the genus level, *5-7N15*, *Oscillospira*, *Roseburia*, *Dorea*, *Preussia*, *Neoascochyta*, *Naganishia*, and *Sporormiella* were enriched in yak feces of different months old. The abundance and proportion of bacteria *Firmicutes*, *Bacteroidetes*, *5-7N15*, and fungi *Mucoromyceta* changed significantly before and after weaning. With the increase of months, *Verrucomicrobia* and *Akkermansia* have shown a downward trend. Through the prediction and analysis of fecal microbial function, it was found that at the level of primary pathways, weaning has a significant impact on cellular processes, environmental information processing, genetic information processing, metabolism, and organismal systems. At the level of secondary metabolic pathways, weaning has a significant impact on cell motility, signal transduction, folding, sorting and degradation, translation, amino acid metabolism, glycan biosynthesis and metabolism, metabolism of terpenoids and polyketides, and xenobiotics biodegradation and metabolism. In addition, by analyzing the differences in functional pathways and microbial composition between sample groups of different months, it was found that the differences in functional pathways were related to the abundance differences of some microorganisms. In general, the changes in the composition and structure of yak fecal microflora may reflect the adaptability of the intestinal microbiota.

## 1. Introduction

Yaks are herbivorous ruminants mainly living in the high mountains with an average altitude of more than 3000 metres, centred on China's Qinghai-Tibetan Plateau. Worldwide, there are approximately 17 million yaks. Approximately 14 million yaks live in China, primarily in Qinghai, Yunnan, Tibet, Gansu, and other provinces (regions) [1]. They are the main source for herdsmen to obtain milk, meat, and other means of livelihood. Yaks have formed special physiological adaptability, nutritional metabolism, foraging characteristics, and special gastrointestinal microbial community to adapt to environmental problems such as plateau, severe cold and hypoxia, and lack of feed.

Animal intestinal microflora is mainly composed of bacteria, fungi, archaea, viruses, and other microorganisms. With the in-depth study of intestinal microbiota, it is found that the host's health is greatly affected by them [2], can provide nutrition for the body, regulates metabolism and intestinal epithelial development, and induces innate immunity [3]. In addition, studies have also proved that intestinal microorganisms are the guarantee for ruminants to digest, feed, establish the immune system, and give play to production performance [4, 5]. Previously, studies have reported the rumen bacterial diversity and the composition and diversity of bacteria in the small intestine and cecum of adult yaks [6]. Weaning is one of the important stages in yak's life. It can not only train calves to eat coarse grain but also stimulate the development of the gastrointestinal tract and enhance their disease resistance to a great extent. However, it is unclear what the composition, diversity, and function pathways of intestinal microorganisms are in the weaning period of yaks.

In light of the importance of intestinal microbiota, we analyzed the composition and diversity of fecal microflora of yaks before and after weaning using 16S rRNA and ITS high-throughput sequencing and predicted microbial functions based on gene composition. This study not only improves our understanding of the microbial composition of yak feces before and after weaning but also provides a reference for the nutritional regulation of yak weaning.

## 2. Methods and Materials

### 2.1. Statement of Animal Ethics

Animal experiments were conducted in compliance with the regulations of the Administration of Affairs Concerning Experimental Animals (Ministry of Science and Technology, China; revised in June 2004). Animal care and management were performed in accordance with regulation and approved by Shihezi University's Bioethics Committee.

### 2.2. Animal Handling and Sampling

A total of 12 healthy yaks in 4 age groups of 3, 4, 5, and 6 months old were selected as the subjects (*n* = 3). Yaks graze freely in the natural pasture (43° 53′ 45.19″ north latitude and 87° 33′ 0.37″ east longitude) with high altitude and cold climate near Urumqi City, Xinjiang Uygur Autonomous Region, weaned at 4 months. Fresh feces of yaks were collected immediately with sterile tubes after they defecate. After the tubes were frozen in liquid nitrogen, they were transported to the laboratory, where they were stored at -80°C until further analysis. The 3-month-old group is group A, the 4-month-old group is group B, the 5-month-old group is group C, and the 6-month-old group is group D.

### 2.3. DNA Extraction

All genomic DNA samples were extracted with Omega DNA Reagent (D5625-01) (OMEGA Biotechnology Ltd., USA, USA) according to the manufacturer's instructions and stored at -20°C. DNA content and quality were determined by the NanoDropND-1000 spectrophotometer (Thermo Fisher Scientific, Waltham, MA, US) and agarose gel electrophoresis.

### 2.4. Amplicon Sequencing

#### 2.4.1. 16S rRNA Gene Sequencing

The primer sequences amplified in the V3-V4 region of bacteria are F 5′-ACTCCTACGGGAGGCAGCA-3′ and R 5′-GGACTACHVGGGTWTCTAAT-3′ [7, 8]. For multiplex sequencing, primers were incorporated with 7-bp barcodes specific to each sample. PCR components included 5 *μ*l of buffer solution (5×), FastPfu DNA polymerase (5 U/*μ*l) 0.25 *μ*l, dNTPs (2.5 *μ*M) 2 *μ*l, 1 *μ*l of forward and reverse primers, DNA template 1 *μ*l, and 14.75 *μ*l of ddH_2_O. PCR reaction conditions were 98°C for 5 minutes, 98°C for 30 seconds, 53°C for 30 seconds, 72°C for 45 seconds, 25 times, and finally 72°C for 5 minutes. PCR amplicons were purified using Vazyme VAHTSTM DNA Clean Beads (Vazyme, Nanjing, China) and quantified using the Quant-iT PicoGreen dsDNA Assay Kit (Invitrogen, Carlsbad, CA, USA). After the quantification step of separation, equal amounts of amplicons were fused and then sequenced with paired-end 2 × 250 bp using the Illumina MiSeq platform with MiSeq Reagent Kit v3 from Shanghai Personal Biotechnology Co., Ltd (Shanghai, China).

#### 2.4.2. Internal Transcribed Spacer (ITS)

The forward primers ITS1F (5′-CTTGGTCATTTAGAGGAAGTAA-3′) and the reverse primer ITS2R (5′-GCTGCGTTCTTCATCGATGC-3′) were used to target amplification of fungal internal transcription (ITS). The PCR components contained buffer solution (5×) 5 *μ*l, 0.25 *μ*l FastPfu DNA Polymerase (5 U/*μ*l), 2 *μ*l dNTPs (2.5 mM), 1 *μ*l of forward and reverse primers (10 *μ*M), 1 *μ*l of DNA Template, and ddH_2_O 14.75 *μ*l. Thermal cycling was an initial denaturation at 98°C for 5 min followed by 28 denaturation, at 98°C for 30 s, annealing at 55°C for 30 s, extension at 72°C for 45 s, and extension at 72°C for 5 min. PCR amplification was performed using the Vazyme VAHTSTM DNA Clean Beads (Vazyme, Nanjing, China) with the Quant-iT PicoGreen dsDNA Assay Kit (Invitrogen, Carlsbad, CA, USA). After individual quantification, Shang Personal Biotechnology Co., Ltd (Shanghai, China), sequenced the 2 × 250 bp sequence using the MiSeq Reagent Kit v3 with Illumina MiSeq platform.

### 2.5. Sequence Analysis

This study adopted QIIME2009.4 [9] and on this basis made some modifications to the formal teaching of microbiota bioinformatics. Briefly, the raw sequence data was processed through the demux plugin, and cutadapt was used for primer cutting. Next, using the DADA2 plugin, the sequences were quality filtered, denoised, merged, and chimeras removed [10]. Non-singleton amplicon sequence variants (ASVs) were obtained by dereplication. Based on the UNITE Release 8.0 databases and SILVA Release 132 [11], the classify-sklearn naïve Bayes taxonomy classifier in feature-classifier plugin [9] was used to assign taxonomies to ASVs.

### 2.6. Predictive Functionality

The PICRUSt2 (Phylogenetic Survey of Reconstructing Communities Using Unobserved States) algorithm software was used to infer the functional profile of a sample from 16S rRNA and ITS marker genes. A new evolutionary tree was established by comparing the representative sequences of 16S rRNA and ITS. Based on the copy number of the gene family corresponding to the reference sequence in the evolutionary tree, we used the castor hidden state prediction algorithm, infer the nearest sequence species of the characteristic sequence, and then obtain the copy number of gene families. The number of copies of each gene in each sample was obtained by analyzing representative sequences from each sample. At last, the gene families were mapped against the KEGG database for bacteria and MetaCyc database for fungi, respectively, and MinPath was used to infer the existence of functional pathways, to obtain the abundance data of functional pathways in each sample at levels 1 and 2.

### 2.7. Bioinformatics and Statistical

The sequence data were analyzed using QIIME2 and the R package (version 3.2.0). An ASV-level rarefaction curve was performed for each sample, and the sequencing depth was analyzed. The R package “VennDiagram” was used to generate Venn diagrams, which can display core and unique ASVs between different groups [12]. The ASV table was used to calculate alpha diversity indices at the ASV level, such as the Chao1, Shannon, Simpson, and Good's coverage, and then analyzed by ANOVA (analysis of variance) through SPSS (version 26.0). The fecal microbiological composition and abundance of each group at the phylum and genus levels were displayed by species classification level annotation, and the analysis results were presented in a histogram, and then the *t*-test between the two groups was carried out by the SPSS software (version 26.0). The linear discriminant analysis effect size (LEfSe) method was used to detect differentially abundant taxa among groups based on the default parameters of the model [13]. Taxa with an LDA (linear discriminant analysis) score > 3 were regarded as important indicators of each group. The ANOVA hypothesis test software was used to statistically analyze the predicted primary functional pathway of bacteria and fungi at levels 1 and levels 2, and the relationships between functional capacity and predicted relative gene abundances were analyzed using heatmaps at level 2. MetagenomeSeq was used to analyze metabolic pathways with significant differences every two groups. Then, according to the metabolic pathway abundance table of the classified samples, the species composition of different pathways was analyzed, and a histogram of the species composition was drawn. Statistical analysis was performed with R and SPSS 26.0. *P* values < 0.05 were considered significant difference.

## 3. Results

### 3.1. Sequence Data

1271872 bacterial original sequences and 1616014 fungal original sequences were obtained from 12 samples. The Dada2 method was used for deprimer, quality filter, denoise, splicing, and dechimaerism, 812033 high-quality bacterial sequences and 1432448 high-quality fungal sequences were obtained, and the numbers of high-quality sequences per sample were 67669 and 119371. After quality control with DaDa2, each weight-removed sequence was ASV (amplification sequence variation). Core ASVs are ASVs observed in each sample. In the bacterial analysis of all samples, we identified 1185 core ASVs, 4040 ASVs unique to group A, 3680 ASVs unique to group B, 3666 ASVs unique to group C, and 4748 ASVs unique to group D (Figure 1(a)). In the fungal analysis, there were 138 core ASVs in all samples, and the specific ASVs in group A, B, C, and D were 294, 464, 383, and 449 (Figure 1(b)). The length of high-quality bacterial sequences contained in the sample was mainly distributed between 404 and 425 bp, and that of fungi was mainly 170-270 bp. To assess whether the sequence ranges we extracted could accurately describe the species composition and relative abundance of each species, sparse curves were drawn based on the Chao1 index and the pumping depth under the sample ASVs (Figures 1(c) and 1(d)). As shown in the chart, the sequencing depth of each sample had basically reached saturation, and the sequencing results were enough to reflect the species diversity of each sample.

### 3.2. Alpha Diversity Analysis

The composition of fecal microbial communities in yak before and after weaning was characterized by the alpha diversity. Good's coverage index [14] represents coverage, Chao1 index [15] represents richness, Shannon index [16] represents equitability, and Simpson index [17] represents diversity. The results showed that the Good's coverage estimations of all sample species range were higher than 97%. The Chao1 index was the lowest in the 4-month-old samples, but it showed an upward trend after weaning. In contrast, the Chao1 index in the fungal community was the highest in the 4-month-old and the lowest in the 3-month-old, and there was significant difference between the two groups (*P* < 0.05). The Shannon and Simpson indices of feces bacteria and fungi were in a fluctuating process with the increase of age before and after weaning, but no significant differences were found among the groups (Table 1).

### 3.3. Bacterial Community Structure

The bacterial phyla with the relative abundance in the top 9 in fecal samples were analyzed (Figure 2(a)). *Firmicutes*, *Bacteroidetes*, and *Verrucomicrobia* were the dominant phyla. The relative abundance of *Firmicutes* ranged from 71.50% to 78.76% (73.08% at 3 months, 78.76% at 4 months, 75.43% at 5 months, and 71.50% at 6 months). It increased significantly from 3 months to 4 months and decreased from 4 to 6 months (Table 2). *Bacteroidetes* was the second dominant phylum, and its relative abundance ranged from 17.92% to 27.80% (3-month-old, 19.94%, 4-month-old 18.57%, 5-month-old 22.76%, and 6-month-old 25.86%). The relative abundance of *Bacteroidetes* at 6 months of age was the highest. Compared with 3 months old, the abundance of 4 months old decreased slightly but increased at 4-6 months old, and there was a significant difference between 4 months old and 5 months old (Table 2). The relative abundance of *Verrucomicrobia* ranged from 0.47% to 4.74%, of which the highest was 4.74% at the age of 3 months before weaning and in other months was less than 1%. Other phyla, such as *Proteobacteria*, *Tenericutes*, *Actinobacteria*, *TM7*, and *Cyanobacteria* were detected. The average relative abundance of each group was less than 0.5%, and the overall expression level was low.

We detected 9 genera in the samples (Figure 2(b)). Of these, *5-7N15*, *Oscillospira*, *Roseburia*, *Dorea*, *Clostridiaceae_Clostridium*, and *Ruminococcaceae_Ruminococcus* were the dominant genera in all age groups. *5-7N15* has the highest abundance, and its relative abundances at 3-6 months old were 7.34%, 3.61%, 5.47%, and 6.83%, of which at 3 months old was the highest and that of 4 months old was the lowest, and the difference between 3 and 4 months old was significant (Table 2). The relative abundance of the strictly anaerobic bacteria *Roseburia* at the age of 3-6 months was 1.13%, 1.25%, 2.29%, and 1.14%. Its relative abundance at 5 months old was higher, at 3-5 months old, it showed an increasing trend, at 5-6 months old, it showed a decreasing trend, and the differences between 3 months old and 5 months old and 5 months old and 6 months old were significant (Table 2). *Oscillospira*, *Dorea*, *Clostridiaceae_Clostridium*, and *Ruminococcaceae_Ruminococcus* were the dominant genera of yaks before and after weaning, and there was no significant difference among the groups. *Akkermansia* is a Gram-negative anaerobic bacterium that is representative of *Verrucomicrobia*. The relative abundance of *Akkermansia* at 3 months before weaning was 4.72% higher than that in other months. Its abundance at other ages was less than 0.8%.

### 3.4. Fungal Community Structure

*Ascomycota* (71.47% at 3 months, 76.44% at 4 months, 77.55% at 5 months, and 76.61% at 6 months) and *Basidiomycota* (7.25% at 3months, 9.05% at 4 months, 4.58% at 5 months, and 9.46% at 6 months) were the most represented phyla in all age groups (Figure 3(a)). The abundance of *Ascomycota* after weaning was higher than that before weaning, and the abundance of *Basidiomycota* was the lowest at 5 months, while there was no significant difference in the relative abundances of *Ascomycota* and *Basidiomycota* among all the groups. The relative abundance of *Mucor*omycota at 6 months (2.16%) was the highest, and less than 1% in other month-old samples. There was a significant difference in the abundance of *Mucor*omycota fungi at the age of 3 and 4 months (Table 3).

The relative abundances of 9 fungal genera were analyzed, and the result showed that the relative abundances of most genera was less than 2.0% (Figure 3). Among the genera with relative abundance more than 2%, *Preussia* (14.17% at 3 months, 18.13% at 4 months, and 22.07% at 5 months) and *Naganishia* (3.24%, 2.60%, 2.39%, and 2.95%, respectively) exist in each month age group and were the dominant genera. *Neoascochyta* was included in those with a relative abundance of more than 2% at the age of 3 months (6.29%), at 4 months of age, including *Pichia* (3.09%). At the age of 6 months, there are more genera with relative abundance of more than 2% than other months, including *Pichia* (24.42%), *Neoascochyta* (4.10%), *Sarocladium* (2.31%), *Mucor*, and *Leucosporidium* (2.45%). According to statistical analysis, there was no significant difference among the dominant fungi (Table 3).

We used the LEfSe analysis to identify the taxa with the strongest differentiation in different month age groups. By comparing with other groups, more differences in bacteria and fungi were found. At the age of 3 months, several microbial populations were enriched at the genus level, including *Akkermansia*. At the age of 4 months, *Cladophialophora* was enriched. Only one genus, *Clostridium*, was found at the age of 5 months. *Filobasidium* and *Leucosporidium* were enriched at the age of 6 months. Interestingly, no fungal biomarkers were found at 3 months of age (Figures 4(a) and 4(b)).

### 3.5. Functional Prediction of Fecal Microbiota Using PICRUSt

The PICRUSt2 analysis was used to predict intestinal bacterial function based on 16S rRNA sequencing data. The results showed that at level 1, the relative abundance of metabolic pathways was the highest, accounting for 77.44%, 76.59%, 77.14%, and 77.29% of the identified pathways in samples aged 3, 4, 5, and 6 months old, respectively, followed by genetic information processing, cellular processes, environmental information processing; functional pathways of organismal systems, and human diseases (Table 4). By comparing the samples among different age groups, it was found that the pathways with differences between 3-month and 4-month age groups were the most common, including cellular processes, environmental information processing, genetic information processing, metabolism, and organismal systems. In addition, there were significant differences in cellular processes, environmental information processing, and metabolism between 4 and 6 months old. And there was a significant difference in environmental information processing between 5 and 6 months old.

A total of 31 biochemical pathways were identified in the second-level pathway, including 11 biochemical pathways of metabolic function. Among them, carbohydrate metabolism, amino acid metabolism, metabolism of cofactors and vitamins, metabolism of terpenoids and polyketides, metabolism of other amino acids, and energy metabolism were highly enriched in all group samples. Additionally, pathways involved in replication and repair, translation, folding, sorting and degradation, and cell motility were predominant in samples from each month of age. Moreover, cell motility, signal transduction, folding, sorting and degradation, translation, amino acid metabolism, glycan biosynthesis and metabolism, metabolism of terpenoids and polyketides, xenobiotics biodegradation, and metabolism were significantly different between 3 and 4 months old. Additionally, there were significant differences in cell motility, signal transmission, glycan biosynthesis, and metabolism between 4 and 6 months old. The abundance of membrane transport pathway in 3-5 months old was higher than that in 6 months old, and there was a significant difference with 6 months old (Table 5).

Using the PICRUSt2 analysis based on the MetaCyc database, we predicted the functional potential of fecal fungi of yaks of different months before and after weaning. This finding shows that the relative abundance of biosynthesis is the highest, accounting for 43.73%, 43.98%, 43.98%, and 44.16% of the identified pathways in the 3-, 4-, 5-, and 6-month-old samples, respectively. In addition, the generation of precursor, metabolite, and energy was also dominant in samples of different age groups, with relative abundances of 36.77%, 36.02%, 36.41%, and 36.11%, respectively (Figure 5(a)). Moreover, there was no significant difference in the main functional pathways among the groups. Among the 29 secondary MetaCyc pathways, the relative abundances of nucleoside and nucleotide biosynthesis, respiration, and electron transfer were the highest in samples of different months old. Additionally, fermentation, TCA cycle, and secondary metabolite biosynthesis pathways were significantly enriched in 3-month-old samples compared to 4-month-old samples (*P* < 0.05). There was a significant difference in amino acid degradation between 3-month-old and 5-month-old samples (Figure 5(b)).

We analyzed the significant differences in functional pathways between the yak groups at each month of age before and after weaning and found that compared with 4 months of age and 3 months of age, GLUCOSE1PMETAB-PWY: glucose and glucose-1-phosphate degradation was significantly down regulated (Figure 6(a)). The species composition of this pathway was analyzed, and the results showed that *Akkermansia* contributed significantly to this pathway (Figure 6(b)). Compared with 5 months old and 4 months old, PWY-7374: 1,4-dihydroxy-6-naphthoate biosynthesis I was significantly upregulated; PWY-6107: chlorosalicylate degradation, P341-PWY: glycolysis V (*Pyrococcus*) and P261-PWY: coenzyme M biosynthesis I were significantly down regulated (Figure 6(c)). Analysis of the species composition of PWY-7374,1,4-dihydroxy-6-naphthoate biosynthesis I and PWY-6107 pathways (Figures 6(d) and 6(e)) revealed *unidentified_Rikenellaceae* has a higher contribution value in the above two pathways. In the P341-PWY pathway, the contribution value of *unidentified_Lachnospiraceae* was higher (Figure 6(f)). There were two differential metabolic pathways between 6-month-old and 5-month-old, among which PWY-7446: sulfoglycolysis was significantly up regulated and PWY-4722: creatinine degradation II was significantly down regulated (Figure 6(g)). In PWY-7446 pathway, *Shigella* and *unclassified_Enterobacteriaceae* played an important role (Figure 6(h)).

## 4. Discussion

In our research, we described the diversity, composition, and potential function of bacteria and fungi in yak fecal before and after weaning based on 16S rRNA and ITS high-throughput sequencing. When searching for shared bacterial and fungi ASVs in all groups, we successfully detected 1185 and 138 ASVs shared ASVs respectively, and each group has its own unique ASVs, which indicated that each group of them contained similar bacterial and fungal communities and was also specific in terms of microbial DNA components. Alpha diversity analysis has shown that the Chao1 index of fecal bacteria of yak decreased first and then increased; this is similar to the study on the composition and changes of intestinal flora in early weaned piglets [18]. However, the Chao1 index of fungi in 4-month-old yaks was higher than that in other months. It is speculated that during weaning, yak diet structure changes, the gastrointestinal microbiota was in the process of dynamic change, and various microorganisms entering the gastrointestinal tract early may be detected. The Shannon index of bacteria and fungi has shown an overall upward trend after weaning, which also indicated an increase in equitability with developmental age. Similar reports were also found in other species, such as pigs, sheep, and horses [19]. However, the Shannon index and Simpson index did not differ significantly among the groups, suggesting that the structure of fecal microflora may dynamically change and tend to become stable with increasing host age.

The results showed that the bacteria in yak feces in different months before and after weaning were mainly *Firmicutes* and *Bacteroides*. Similarly, *Firmicutes* and *Bacteroidetes* are also mentioned as the two main phyla in a study of human intestinal flora [20] and in the composition and structure of microbial community in forest musk deer feces [21]. In this study, the abundance of *Firmicutes* decreased, while *Bacteroides* increased after weaning, which may be related to the change in the yak diet structure from milk and natural forage with high animal protein, fat, and carbohydrate to natural forage with high fiber. Some scholars have suggested that the number of *Bacteroides* was found to be lower in children fed a high-calorie diet. When a high-fiber diet was introduced, the content of *Bacteroides* was higher and that of *Firmicutes* was lower [22], which is consistent with our research results. Both *Firmicutes* and *Bacteroides* are responsible for the digestion of carbohydrates and proteins. It is speculated that the high abundance of *Firmicutes* and *Bacteroides* in yak feces before and after weaning is related to the high energy consumption of yaks living at high altitude [23]. *Firmicutes* can also regulate the immune response in vivo, inhibit the invasion of pathogens, and prevent intestinal inflammation [21], which also shows that there is a mutually beneficial symbiotic relationship between intestinal microorganisms and the host. This research demonstrated that the abundance of *Verrucomicrobia* in fecal samples before weaning was higher than that after weaning, which was related to the host's diet and physiological condition. Studies have shown that the low abundance of *Verrucomicrobia* was related to the increase of fiber intake [24]. The fiber intake of yaks after weaning was higher than that before weaning, so this phylum has shown a decreasing trend after weaning. Other phyla, such as *Tenericutes*, *Actinobacteria*, *TM7*, and *Cyanobacteria*, were detected in feces from 3 months to 6 months old, but the overall proportion was small. However, they were also important components of the intestinal microbial diversity of yaks before and after weaning.

There were a large number of unclassified bacteria at the genus level, which was similar to the previous studies results on yak rumen microbial diversity, indicating that further exploration of yak intestinal microorganisms and their functions is necessary. It was reported that *5-7N15* was the dominant genus in musk deer [25] and Hainan Polu [26], and *5-7N15* had a significant positive correlation with the crude fiber digestibility [27]. The high abundance of *5-7N15* in this study may be related to the feeding of yaks with natural forage containing a large amount of crude fiber. The relative abundance of *Akkermansia* at the age of 3 months was higher than that of other months. Similarly, some studies have proved that this bacterium was also found in 3-day-old and 42-day-old calves [28]. In addition, *Akkermansia* plays an active role in maintaining the internal mucosal barrier and anti-inflammatory. It is inferred that this bacterium does play key roles in reducing the occurrence of intestinal diseases during yak weaning.

Most of the bacteria initially colonized in the intestine are aerobic or facultative anaerobic bacteria. With the increase of months, the intestinal anaerobic environment was formed, including the abundance of anaerobic bacteria *Roseburia*, *Oscillospira*, Clostridium, and *Ruminococcus* that increased and tended to be stable. In addition, *Roseburia*, *Clostridium*, and *Ruminococcus* are the core flora producing short chain fatty acids and play a vital role in maintaining intestinal health, such as regulating intestinal pH and mucus production, providing energy for epithelial cells and affecting mucosal immune function to maintain intestinal integrity [29, 30]. It is speculated that this may enhance the body's resistance to diseases to a certain extent.

In our results, *Ascomycota* and *Basidiomycota* were the most abundant phyla in the yak fecal fungal community, and the sum of the average abundance of the two phyla in 3-month-old yak feces had reached more than 75%, which is consistent with the research results of herbivorous ruminants such as cattle [31] and sheep [32]. At the same time, t was found that these two are also the main phyla of cellulose degradation [33], which can provide various nutrients for the host. *Mucor*omycota was also the dominant fungus before and after weaning. It is a widespread saprophytic fungus with efficient lignin decomposition function. Studies have proved that it also widely exists in the gastrointestinal tract of beef cattle [34]. However, some studies have pointed out that under grazing feeding mode, this fungus exists only in a small amount in adult tan sheep, but not in the shed-feeding group [35]. The abundance of this fungus was significantly higher at 4 months than at 3 months old. This may be related to the fact that the fungus is greatly affected by dietary structure, external environment, and other factors. The relative abundance of *Mortierellomycota* increased with the increase of months, and there was a significant difference between 3 and 5 months. Previous studies have shown that *Mortierellomycota* is negatively correlated with age [36], which is different from our results, which also confirms the view that intestinal microorganisms are affected by many factors.

The results of this study showed that *Preussia* was the genus with the highest abundance in yak feces in different months, which is consistent with the results of cattle and yaks living on the plateau without supplementary feeding in winter [31]. It is reported that *Preussia* has good antibacterial capacity [37] and antioxidant capacity [38]. We found that *Preussia* abundance has shown an increasing trend with the increase of months, which may indicate that yak disease resistance, immune system development, and environmental adapt ability are gradually enhanced with the increase of age. *Pichia* can well express foreign proteins [39] and effectively inhibit Candida infection. This study found that *Pichia* has shown an upward trend after weaning, which may improve the disease resistance and anti-inflammatory properties of yaks and promote the improvement of immune response system. These data have shown that with the growth of yak age, intestinal microorganisms become increasingly complex and disease resistance becomes stronger and stronger.

PICRUSt functional prediction analysis showed that the functional genes of yak fecal bacterial at different ages were most enriched in the metabolic pathway, while the functional genes of fungi were the most abundant in biosynthesis and generation of precursor metabolites and energy, reflecting that intestinal microorganisms would help the host improve energy utilization efficiency and adapt to the high energy consumption environment at high altitude. In the month of weaning (4 months old), the functional pathways of cellular processes, environmental information processing, genetic information processing, metabolism, and organismal systems were significantly different from those before weaning (3 months old), indicating that weaning has a significant impact on the potential function of bacteria at level 1. At level 2, glycan biosynthesis and metabolism, xenobiotics, biodegradation, and metabolism were more enriched in before weaning yaks at 3 months old, while folding, sorting and degradation, translation, amino acid metabolism, metabolism of terpenoids and polyketides, and amino acid degradation were more enriched in the after weaning yaks (4-6 months old), and cell mobility and signal translation were enriched at 4 months old, indicating that the host was in different growth stages; the function of intestinal microorganisms will change to help the host better adapt to the living environment. Among the secondary functional pathways, 22 KEGG pathways and 26 MetaCyc pathways have no significant difference, which indicates that weaning has different effects on the potential function of intestinal microorganisms, which may be related to the differences in the adaptation of yak intestinal microbiota to external environmental changes.

We analyzed the significantly different functional pathways and the species composition of pathways between the sample groups of different months and found that the differences of functional pathways were related to the differences of some species. The characteristic microorganisms of different age groups affect the functional pathways to adapt to the changes of the external environment. In addition, in the species composition of some significant difference paths, the genera with large contribution values have not been classified, such as *unidentified ones_Rikenelaceae*, *unidentified_Lachnospiraceae*, and *unclassified_Enterobacteriaceae*, showing that there are a large number of unknown microorganisms in yak feces. How they participate in important physiological processes such as metabolism, nutrition, and immunity remains to be further studied.

## 5. Conclusions

In conclusion, we used 16S rRNA and ITS high-throughput sequencing to study and prove the dynamic distribution of fecal microbial community development of yaks at different months before and after weaning. The potential functions of yak fecal microbiota were analyzed by PICRUSt. The results showed that weaning has a significant impact on the richness of fecal fungi but had no significant influence on the diversity and equitability of fecal bacteria and fungi. The abundance and proportion of some fecal microorganisms changed significantly before and after weaning, including bacteria *Firmicutes*, *Bacteroidetes*, *5-7N15*, and fungus *Mucoromyceta*. With the increase of months, the relative abundance of *Firmicutes* decreased, while the relative abundance of *Bacteroidetes* and *Mucor*omycota increased. Weaning changed the expression of genes involved in Cellular Processes, information processing, and nutrient metabolism in fecal microorganisms. In addition, some unclassified microorganisms play an important role in functional pathways. Therefore, it is necessary to further excavate yak intestinal microorganisms and evaluate their effects on physiological functions. This study can provide an important theoretical basis for microbiota-based treatment or disease prevention strategies.

## Figures and Tables

**Figure 1:** Fecal microbial amplicon sequence variants (ASVs) in different months. (a) Bacterial Venn diagram, where the overlapping area represents the number of ASVs shared between overlapping groups. (b) Fungal Venn diagram. (c) Bacteria rarefaction curves for each sample. (d) Fungal rarefaction curves for each sample. A: at 3 months; B: at 4 months; C: at 5 months; and D: at 6 months.

**Figure 2:** The composition of fecal bacteria in yaks of different months at phylum and genus levels. (a) Relative abundance of different phylum in samples of different months. (b) Relative abundance of different genus in samples of different months.

**Figure 3:** The composition of fecal fungal in yaks of different months at phylum and genus levels. (a) Relative abundance of different phyla in samples of different months. (b) Relative abundance of different genus in samples of different months.

**Figure 4:** Histogram showing taxa with statistically significantly LDA values of yaks at different ages. (a) LEfSe analysis of fecal bacterial communities. (b) LEfSe analysis of fecal fungal communities. f: family; g: genus; s: species; o: order.

**Figure 5:** Prediction of potential functions of fecal fungi from yaks of different ages. (a) Predictive functional components (%) of fecal fungi in yaks of different months of age at level 1. (b) Predictive functional components (%) of fecal fungi in yaks of different months of age at level 2.

**Figure 6:** Analysis of different functional pathways and species composition of yaks in different months. (a) Analysis of metabolic pathways in 4-month-old and 3-month-old yaks. (b) Species composition of GLUCOSE1PMETAB-PWY, glucose, and glucose-1-phosphate. (c) Analysis of metabolic pathways in 5-month-old and 4-month-old yaks. (d) Species composition of PWY-7374,1,4-dihydroxy-6-naphthoate biosynthesis I. (e) Species composition of PWY-6107 chlorosalicylate degradation. (f) Species composition of P341-PWY glycolysis V (*Pyrococcus*). (g) Analysis of metabolic pathways in 6-month-old and 5-month-old yaks. (h) Species composition of PWY-7446 sulfoglycolysis.

**Table 1:** Alpha diversity indices of yak fecal microbial community in different months before and after weaning.

Treatments	Bacterial community^1^				Fungal community^1^			
	Good's Chao1 Shannon Simpson				Good's Chao1 Shannon Simpson			
3-month-old	0.9799 ± 0.0054	3635.53 ± 494.70	9.84 ± 0.21	1.00 ± 0.00	1.0000 ± 0.0000	285.06 ± 27.06^a^	5.02 ± 0.17	0.92 ± 0.00
4-month-old	0.9818 ± 0.0017	3469.79 ± 72.36	10.00 ± 0.15	1.00 ± 0.00	0.9999 ± 0.0000	419.39 ± 12.16^b^	5.49 ± 0.23	0.94 ± 0.01
5-month-old	0.9793 ± 0.0025	3615.05 ± 398.76	9.87 ± 0.21	1.00 ± 0.00	0.9999 ± 0.0000	351.73 ± 33.75^ab^	5.03 ± 0.10	0.92 ± 0.01
6-month-old	0.9823 ± 0.0062	3635.08 ± 701.26	10.05 ± 0.22	1.00 ± 0.00	0.9998 ± 0.0001	355.59 ± 44.79^ab^	5.26 ± 0.58	0.91 ± 0.03

^1^Comparisons between different months of age groups based on a multivariate analysis of variance (ANOVA). The values were presented as the mean ± SEM; SEM: standard error of mean. In the same column, there is no letter or superscript with the same letter, the difference is not significant (*P* > 0.05), while in different lowercase letters, there is a significant difference (*P* < 0.05).

**Table 2:** Taxonomic analysis of the main fecal bacteria, phyla, and genera of yaks, classified according to the time point.

Phylum	Experimental treatments				SEM^1^	*P* value
	3-month-old	4-month-old	5-month-old	6-month-old		
*Firmicutes*	73.08^a^	78.76^b^	75.43^ab^	71.50^ab^	0.88	0.004
*Bacteroidetes*	19.94^b^	18.57^b^	22.76^a^	25.86^a^	0.87	0.001
*Verrucomicrobia*	4.74	0.79	0.47	0.67	0.62	0.023
*Proteobacteria*	0.77	0.54	0.26	0.44	0.09	0.293
*Tenericutes*	0.34	0.40	0.30	0.39	0.04	0.873
*Actinobacteria*	0.39	0.30	0.225	0.26	0.04	0.440
*TM7*	0.15	0.27	0.23	0.35	0.05	0.607
*Cyanobacteria*	0.29	0.11	0.10	0.20	0.03	0.071
Elusimicrobia	0.01	0.02	0.01	0.08	0.01	0.068
Genus						
*5-7N15*	7.34^a^	3.61^b^	5.47^ab^	6.83^ab^	0.68	0.269
*Oscillospira*	3.91	4.13	4.78	4.22	0.17	0.418
*Akkermansia*	4.72	0.73	0.43	0.56	0.63	0.02
*Roseburia*	1.13	1.25	2.29	1.14	0.21	0.196
*Dorea*	1.23	1.10	2.23	1.06	0.23	0.263
*Clostridiaceae_Clostridium*	0.77	1.43	1.34	1.47	0.17	0.529
*Ruminococcaceae_Ruminococcus*	0.75	0.91	0.85	1.12	0.11	0.757
CF231	1.59	0.16	0.27	1.06	0.38	0.606
SMB53	1.03^a^	0.85^a^	0.69^a^	0.16^b^	0.12	0.033

^1^SEM: standard error of mean. ^a,b^In the same line, there were significant differences in values of different superscripts (*P* < 0.05).

**Table 3:** Taxonomic analysis of the main fecal fungal phyla and genera of yaks, classified according to the time point.

Phylum	Experimental treatments				SEM	*P* value
	3-month-old	4-month-old	5-month-old	6-month-old		
*Ascomycota*	71.47	76.44	77.55	76.61	2.65	0.899
*Basidiomycota*	7.25	9.05	4.58	9.46	1.03	0.411
*Mucor*omycota	0.14^a^	0.54^b^	0.34^ab^	2.16^ab^	0.44	0.446
Neocallimastigomycota	0.03	0.50	0.40	0.20	0.09	0.345
Mortierellomycota	0.05	0.43	0.45	0.10	0.08	0.211
Genus						
*Preussia*	14.17	18.13	22.07	11.54	1.65	0.128
*Pichia*	0.33	3.09	0.36	24.42	4.35	0.170
*Neoascochyta*	6.29	1.49	1.74	4.10	1.31	0.631
*Naganishia*	3.24	2.60	2.39	2.95	0.52	0.963
*Sporormiella*	1.23	1.47	1.79	1.29	0.29	0.936
*Sarocladium*	0.45	1.41	1.21	2.31	0.51	0.729
Aspergillus	0.53	0.98	0.71	0.89	0.12	0.627
Podospora	0.26	1.11	1.15	0.40	0.17	0.165
*Mucor*	0.11	0.33	0.31	2.13	0.45	0.436

^1^SEM: standard error of mean. ^a,b,c^In the same row, values with different letter superscripts mean significant difference (*P* < 0.05).

**Table 4:** Prediction of bacterial functional components (%) in feces of yaks of different age at level 1.

Functions	3-month-old	4-month-old	5-month-old	6-month-old
Cellular processes	5.19 ± 0.12^b^	5.60 ± 0.04^a^	5.27 ± 0.33^ab^	5.24 ± 0.05^b^
Environmental information processing	1.96 ± 0.01^c^	2.00 ± 0.02^a^	1.98 ± 0.05^ac^	1.87 ± 0.02^b^
Genetic information processing	14.75 ± 0.16^b^	15.14 ± 0.11^a^	14.93 ± 0.29^ab^	14.94 ± 0.2^ab^
Human diseases	0.19 ± 0.00	0.19 ± 0.01	0.19 ± 0.01	0.18 ± 0.01
Metabolism	77.44 ± 0.28^a^	76.59 ± 0.07^b^	77.14 ± 0.57^ab^	77.29 ± 0.23^a^
Organismal systems	0.47 ± 0.00^b^	0.48 ± 0.01^a^	0.48 ± 0.01^ab^	0.47 ± 0.00^ab^

^a,b,c^In the same row, values with different letter superscripts mean significant difference (*P* < 0.05). The values were presented as the mean ± SEM; SEM: standard error of mean.

**Table 5:** Prediction of bacterial functional components (%) in feces of yaks of different age at level 2.

Functions	3-month-old	4-month-old	5-month-old	6-month-old
Cellular processes				
Cell growth and death	1.54 ± 0.02	1.56 ± 0.03	1.57 ± 0.01	1.56 ± 0.02
Cell motility	3.27 ± 0.10^b^	3.65 ± 0.08^a^	3.3 ± 0.38^ab^	3.25 ± 0.09^b^
Cellular community, prokaryotes	0.20 ± 0.01	0.20 ± 0.01	0.20 ± 0.01	0.20 ± 0.00
Transport and catabolism	0.18 ± 0.01	0.19 ± 0.03	0.21 ± 0.05	0.23 ± 0.05
Environmental information processing				
Membrane transport	1.58 ± 0.01^a^	1.59 ± 0.01^a^	1.59 ± 0.06^a^	1.49 ± 0.02^b^
Signal transduction	0.39 ± 0.01^b^	0.41 ± 0.01^a^	0.39 ± 0.01^ab^	0.38 ± 0.00^b^
Signaling molecules and interaction	0.00 ± 0.00	0.00 ± 0.00	0.00 ± 0.00	0.00 ± 0.00
Genetic information processing				
Folding, sorting and degradation	3.42 ± 0.03^b^	3.50 ± 0.02^a^	3.43 ± 0.06^ab^	3.45 ± 0.06^ab^
Replication and repair	6.35 ± 0.76	6.50 ± 0.66	6.45 ± 0.09	6.43 ± 0.08
Transcription	1.37 ± 0.02	1.43 ± 0.02	1.39 ± 0.07	1.39 ± 0.01
Translation	3.61 ± 0.05^b^	3.70 ± 0.05^a^	3.66 ± 0.06^ab^	3.66 ± 0.06^ab^
Human diseases				
Cardiovascular diseases	0.00 ± 0.00	0.00 ± 0.00	0.00 ± 0.00	0.00 ± 0.00
Immune diseases	0.00 ± 0.00	0.00 ± 0.00	0.00 ± 0.00	0.00 ± 0.00
Infectious diseases	0.19 ± 0.00	0.19 ± 0.01	0.019 ± 0.01	0.018 ± 0.01
Neurodegenerative diseases	0.00 ± 0.00	0.00 ± 0.00	0.00 ± 0.00	0.00 ± 0.01
Metabolism				
Amino acid metabolism	13.08 ± 0.11^b^	13.45 ± 0.12^a^	13.26 ± 0.25^ab^	13.35 ± 0.24^ab^
Biosynthesis of other secondary metabolites	1.97 ± 0.01	1.98 ± 0.01	1.99 ± 0.02	2.02 ± 0.05
Carbohydrate metabolism	13.32 ± 0.07	13.42 ± 0.08	13.44 ± 0.07	13.34 ± 0.18
Energy metabolism	5.44 ± 0.29	5.31 ± 0.29	5.30 ± 0.31	5.18 ± 0.10
Glycan biosynthesis and metabolism	3.90 ± 0.03^a^	3.44 ± 0.03^b^	3.76 ± 0.25^ab^	3.9 ± 0.12^a^
Lipid metabolism	5.58 ± 0.08	5.55 ± 0.16	5.67 ± 0.12	5.56 ± 0.18
Metabolism of cofactors and vitamins	12.76 ± 0.05	12.80 ± 0.06	12.72 ± 0.08	12.86 ± 0.20
Metabolism of other amino acids	6.78 ± 0.39	6.71 ± 0.05	6.63 ± 0.05	6.91 ± 0.31
Metabolism of terpenoids and polyketides	9.80 ± 0.09^b^	10.23 ± 0.17^a^	10.10 ± 0.30^ab^	10.20 ± 0.35^ab^
Nucleotide metabolism	2.09 ± 0.02	2.12 ± 0.02	2.11 ± 0.01	2.11 ± 0.03
Xenobiotics biodegradation and metabolism	2.71 ± 0.10^a^	1.61 ± 0.21^b^	2.17 ± 1.00^ab^	1.88 ± 1.06^ab^
Organismal systems				
Digestive system	0.03 ± 0.00	0.03 ± 0.00	0.03 ± 0.00	0.04 ± 0.01
Endocrine system	0.10 ± 0.00	0.11 ± 0.01	0.11 ± 0.01	0.10 ± 0.00
Environmental adaptation	0.25 ± 0.00	0.26 ± 0.01	0.26 ± 0.01	0.24 ± 0.01
Excretory system	0.00 ± 0.00	0.00 ± 0.00	0.00 ± 0.00	0.00 ± 0.00
Immune system	0.09 ± 0.01	0.09 ± 0.00	0.09 ± 0.01	0.09 ± 0.00

The values were presented as the mean ± SEM; SEM: standard error of mean. Letters a and b indicate significant differences within the same row (*P* < 0.05).

## Data Availability

The data used to support the findings of this study are available from the corresponding author upon request.
